# Research on Sustainable Development of Transport Infrastructure Based on Corporate Culture and Low-Carbon Perspective

**DOI:** 10.1155/2022/4629422

**Published:** 2022-08-31

**Authors:** Wenbin Fang, Chongsen Ma, Zeyang Lei

**Affiliations:** ^1^Changsha University of Science and Technology, Changsha, Hunan 410000, China; ^2^School of Traffic & Transportation Engineering, Changsha University of Science and Technology, Changsha, Hunan 410000, China

## Abstract

Excellence in corporate culture is the key to achieving sustainable business development. Sustainability can be a source of success, innovation and profitability for a company, driving the achievement of low-carbon goals for transport infrastructure enterprises. The aim of this study is to examine the relationship between corporate culture and corporate sustainability from the perspective of transport infrastructure enterprises, and to identify which corporate culture factors may have an impact on the sustainable low carbon development of transport infrastructure enterprises. To achieve this, we constructed a structural equation model based on 351 cases in Hunan Province and examined the relationship between corporate culture and sustainable low-carbon development using partial least squares structural equation modeling. The findings suggest that corporate values and corporate culture management capabilities play an important role in promoting sustainable development of transport infrastructure enterprises at the economic and low-carbon levels.

## 1. Introduction

The rapid growth of the global population and the demand for transport infrastructure has shown that low-carbon sustainable development of transport infrastructure cannot be achieved by following old development models [1, 2]. At the same time, many researchers now agree that sustainable development cannot be achieved without the sustainable development of business organizations and their cultures [3, 4]. Meanwhile, the 2030 Agenda for Sustainable Development, approved by the United Nations in 2015, establishes 17 Sustainable Development Goals (SDGs), which clearly state that infrastructure has a significant impact on the environment and public health and that improving the sustainability of infrastructure is essential for achieving global sustainable development. Achieving sustainable infrastructure plays a vital role in promoting resource conservation and building the environmental impact of infrastructure, and developing sustainable infrastructure is a crucial way to achieve SDGs 2030 [5, 6].

There is a large body of research on corporate culture, but the definition of culture in existing research is still unclear. Researchers usually consider corporate culture to be “the way we do things around here” [7]. Some scholars have further extended the definition of organizational culture on this basis [8]. It further defines culture as having three levels and states that the values of the users are an important part of the culture.

Meanwhile, in recent years corporate sustainability and sustainable management have become important concerns for the business community [9–12]. In order to achieve sustainable corporate development, researchers have conducted in-depth studies on sustainability strategies, business sustainability, sustainable low-carbon development, and sustainability of organizational management models [13–17]. The results of the study show that companies need to make changes at the corporate culture level in order to achieve their own sustainability. However, transport infrastructure is difficult to achieve sustainable low-carbon development due to its own attributes [18].

Further, the question arises that how exactly does corporate culture impact the risks in sustainable operations in transport infrastructure companies in achieving sustainable low carbon operations? While Arnold's research suggests that individuals play an essential role in the sustainability of a business, Aisma notes that sustainability needs to be based on the cultural attributes of the people in the business. Therefore, a company's culture and ability to manage it are crucial to sustainable development. [19].

In this context, this study aims to answer how does corporate culture contribute to sustainable low-carbon operations in companies?

The current studies are less focused on transportation infrastructure, especially on the impact of sustainable culture and sustainable strategy of transportation infrastructure enterprises on their sustainable development. Therefore, it is of great theoretical and practical significance to research sustainable low-carbon operational factors of transportation infrastructure.

Section 2 presents the current state of research on the concepts of sustainable low carbon operations, operational corporate culture, corporate values, and sustainable operational risk.  Section 3 constructs the research model and describes the scope of the data collection. Section four presents the calculations for the model. The conclusions, shortcomings, and possible future research directions of the study are discussed in Parts 5 and 6.

## 2. Hypothesis and Conceptual Model Development

### 2.1. Sustainable Low-Carbon Operation

The sustainable low-carbon operation of transport infrastructure depends on the relevant capabilities of the enterprise and the industry, through the literature, this study extracts that green dynamic capabilities, green product development, green creativity, and carbon reduction capacity have a direct impact on the sustainable low-carbon operation.

Dynamic capability refers to the use of existing green resources and capabilities to build and develop new organizational capabilities to help companies respond to changing industry environments and meet competitive market demands [20].

Chen and Chang have developed the concept of green dynamic capabilities based on existing research: the ability of a company to use its existing resources and knowledge to update and develop its green organizational capabilities to respond to dynamic markets and conclude that green dynamic capabilities have a positive impact on green innovation and facilitate the development of green products [21].

The efficiency, availability, and sustainability of green product development and its effectiveness once put into use can directly influence our assessment of the level of sustainable low carbon operation in the industry, whether it is a company or an industry. For this reason, this study defines green product development as “research into the application of products that have a low impact on the environment and human health, are easy to recycle in components or as a whole, and consume relatively little energy.” Many research works have shown that green practices such as investing in emission abatement technologies, using recyclable materials, and promoting energy-saving products could significantly drive the market demand [22–25].

Green product development is affected by market demand, and enterprises adjust product development through their own dynamic capabilities, that is, green products with clear and precise purpose will make sustainable and low-carbon operation effective and recover costs more quickly; On the contrary, not paying attention to green product development can easily lead to product development costs that cannot be recovered as planned. Therefore, green product development is an important factor affecting sustainable and low-carbon operations.

Unlike green product development, green innovation is not limited to technological advances and innovations in corporate concepts, green culture, management models, and codes of practice. As an integral part of green supply chain management, green innovation has also received attention in research to promote the development of supply chains in green blocks [26]. By embracing sustainable innovation practices, companies can cut down on adverse social and environmental consequences that are derived from their operations [27].

As part of the traditional industry, transport infrastructure has a mature construction model, but there are still gaps in how enterprises and the industry operate under the theme of sustainable low-carbon operation, how to complete the transition to low-carbon operation while ensuring economic efficiency and market dynamism, and how to propose professional codes of practice for low-carbon requirements.

The ability to reduce carbon emissions is an intuitive indicator to evaluate the level of sustainable low-carbon operation in the industry, and current research is more advanced in measuring carbon emissions. As we know, reducing carbon emissions has a negative impact on the potential capacity output given the current technical level [28]. However, most of the research on carbon emission reduction capacity on the sustainable development of enterprises is focused on the technical and economic aspects, but less consideration has been given to the interaction between the carbon emission reduction capacity of enterprises and corporate culture, i.e., whether enterprises have made carbon emission reduction awareness a priority in the construction of corporate culture, and what role the carbon emission reduction capacity of enterprises has on the construction of low-carbon corporate culture [29, 30].

### 2.2. Sustainable Low-Carbon Operation

Operational corporate culture refers to the elements of a company's code of conduct, operating philosophy, and the management of culture that exist in the course of its operations. This study divides operational corporate culture into two components—corporate culture management capabilities and corporate values.

The main tasks of culture management are the four blocks of culture innovation, migration, implementation, and daily construction management; therefore, we evaluate the enterprise culture management capability in terms of four indicators—culture innovation, culture migration, culture acceptance willingness, and culture management mode.

The first thing that needs to be transformed in transport infrastructure construction enterprises from the past mode of operation that focused on quality, efficiency, and economic benefits to sustainable low-carbon operation is the ideology of the entire enterprise, so building new corporate culture content based on the good traditions of the enterprise becomes an important part of corporate culture management. Differently from product innovation, which is associated with altering the product radically or incrementally, cultural innovation is associated with altering the cultural significance of the product (and of its consumption) according to the cultural needs of target consumers [31].

Therefore, this study uses cultural innovation as one of the indicators to evaluate the capability of corporate culture management.

With the development of transport infrastructure and the frequent crossover of disciplines, the cultural characteristics of the industry itself will be influenced by other disciplines in other industries in the process. However, such a cultural shift does not necessarily fit the needs of the sustainable low-carbon operation, so companies and the industry need to proactively manage the cultural shift in order to adapt to the development direction of sustainable low-carbon operation.

The effectiveness of the cultural management model adopted in the process of cultural construction and management directly affects the efficiency of cultural management. An efficient cultural management model can lead to the rapid acceptance of corporate culture by employees, who are actively engaged in cultural innovation, and cultural migration and thus facilitate the recovery of capital and the creation of economic benefits; conversely, an inefficient cultural management model can hinder these processes. In addition, the cultural management model determines the tendency of corporate culture innovation, cultural migration, and acceptance of new knowledge and information, and plays an important role in the current era of rapid development of themes such as green sustainability.

The willingness to accept different cultures varies across the company and the industry as a whole, especially when the operating model changes and the capital investment causes the stakeholders to have a different view of the company's development. If the enterprise collective fails to reach different opinions on corporate culture and strategy, the sustainable and low-carbon operation is undoubtedly difficult to develop in such an internal environment.

For this reason, this study uses the willingness to accept culture as one of the indicators to measure the ability to manage culture in an organization.

In summary, the following hypotheses were formulated for this study.

  Ha1: Corporate cultural management competencies have a positive effect on sustainable low-carbon operations.
  Ha2: Corporate cultural management competencies have a positive effect on sustainable economic effects.

### 2.3. Corporate Values

At this stage, China is promoting the concept of ecological civilization, which means improving the ecological environment at the level of values. In the same way, the sustainable low-carbon operation needs to be reflected in corporate values.

The purpose of the sustainable low-carbon operation is to protect the ecological environment and resources, which is essentially a social responsibility. Therefore, whether a company takes the concept of sustainable low-carbon operation as its active social responsibility or whether it is willing to take the relevant responsibility reflects its operational corporate culture.

Because of the macro and micro particularities in these Emerging markets, companies tend to disregard vital issues that could improve social and environmental conditions for citizens [32]. In addition, Obada and Dabija found that social media streaming was an intermediary for sharing fake news about environmental brands on social media and that society gave feedback on and spread the corporate brand image [33]. Cătălina et al. pointed out that large companies operating in the Romanian market are familiar with the concept of CSR, but their perspective of CSP varies significantly in terms of the practices and factors of influence considered [34]. Baolong concludes that CSR practices significantly contribute to green innovation, and based on this, this study hypothesizes that social responsibility contributes to sustainable low-carbon operations [35]. Chen's study shows that investing resources to improve green brand image, green satisfaction, and green trust contributes to green brand equity. Based on this, this study hypothesizes that social responsibility contributes to sustainable low-carbon operations [36].

Social responsibility affects the perception of the company in the external environment, while the consistency of values affects the recognition of culture within the company. Values consistency refers to whether companies agree on the values of sustainable low-carbon operations. Values consistency directly affects whether companies can effectively implement the values they have set to drive the development and improvement of sustainable low-carbon operations and reduce the difficulty of sustainable operational governance. At the same time, values consistency also reflects whether corporate values are widely accepted. Companies can improve sustainability by motivating employees, building clear communication, building awareness, and integrating them into the company's strategy [37]. These methods can improve the consistency of corporate values within the enterprise, which in turn affects the sustainability of the enterprise, so this study uses the consistency of values as one of the indicators for evaluating corporate values.

Innovation orientation mainly reflects the degree to which firms are active in innovation, i.e. there is an active innovation orientation and a passive innovation orientation. Active innovation-oriented companies are happy to invest in innovation in the sustainable low carbon sector, actively developing and putting it into use; passive innovation-oriented companies are either constrained by funding or due to their size, do not tend to invest capital in innovation, but are driven by policy, industry environment or difficulties at work. In their study, Chen et al. found that actively generated green ideas play a key role in achieving good green product development performance in firms; whereas reactive green innovations have no significant impact on green innovation and green product development performance [38]. And innovative sharing strategies provide the highest profits for businesses, while individual development strategies produce the lowest profits. The key to competitive advantage begins by defining and then communicating a clear, shared, and integrated vision [39].

On this basis, innovation orientation reflects the motivation of firms to develop sustainable low-carbon operations.

In summary, this study makes the following hypotheses.

  Hb1: Corporate values have a positive effect on sustainable low-carbon operations.
  Hb2: corporate values have a positive effect on the governance of sustainable operations.
  Hb3: There is a positive effect of corporate values on corporate culture management capability.

### 2.4. Sustainable Low-Carbon Operation

Sustainable operation risk mainly comes from the governance of the economy and operations. Economic benefits are the basis for sustainable low carbon operation, and the governance of the operation of the new model affects the economic benefits on the one hand and the effectiveness of sustainable low carbon operation on the other.

The development of sustainable low carbon operation requires stable economic support, and economic benefits depend on various aspects such as the market, policy environment, inputs, and benefits; therefore, the above four aspects need to be integrated when measuring sustainable economic effects.

Low-carbon behavior is different from the behavioral patterns of transport infrastructure in the past, and the promotion of low-carbon behavior requires capital investment and resources, so market feedback is particularly important. Deepak Kumar Srivastava et al. highlight the fact that socioeconomic factors in the workplace are essential for the successful adoption of Industry 4.0 technologies [40]. If there is a general market preference for low carbon behavior, there will be more scope for sustainable low carbon operation and the payback period will be shorter; conversely, if the market preference is not favorable, this will mean that it will be more difficult to pay back the investment and companies will need to change their operating strategies quickly.

The promotion of sustainable low-carbon operation stems from the orientation of the policy environment. In addition, enterprises need to make economic and resource investments in response to policies such as low-carbon development and carbon emission reduction, which will affect the production capacity of enterprises [28]. Therefore, the level of government subsidies in terms of economics and policies will directly influence the motivation of enterprises to transform when they do this.

Sustainable low carbon operation is not limited to being friendly to the environment but is also reflected in the health sustainability of the business, i.e., the business has a degree of savings in sustainable low carbon operation compared to the past mode of operation, which contributes to the economic situation of the business. In the short term, enterprises need to inject capital to change their operating model, and at the same time, the change of the inherent model will reduce the production capacity of enterprises in a short period of time, and if sustainable low-carbon operation lacks long-term investment value, it will be difficult to attract the transformation of enterprises.

Green transition inputs are the “entry barrier” to sustainable low-carbon operations. Companies should integrate sustainability models into their operational processes and optimize their financial data to support operability. Enterprises attempt to subsidize climate adjustment, but their investment decisions are limited by risk profiles related to climate adjustment undertakings, the shortage of financially feasible and bankable operations, and extensive indications of climate risk that shape adjustment decisions [41]. Therefore, reasonable input costs can help to attract more companies to adopt low carbon behavior and make a positive transition towards sustainable low carbon operations.

In summary, this study makes the following assumptions.

  Hc: Sustainable economic effects have a positive effect on sustainable low-carbon operations.

### 2.5. Sustainable Operational Governance

Operational governance generally depends on the level of corporate management and is therefore susceptible to the influence of corporate values, while the level of operational governance has a direct impact on the economic impact of sustainable low-carbon operations. Sustainability, in turn, subsumes three core interlinked pillars in the form of economic, environmental, and social factors [42]. Upadhyay et al. have already established that sustainability is a core focus of the circular economy [43]. Therefore, the efficiency of sustainable operational governance is the key to balancing the economy, the environment, and society.

There are commonalities and differences between the governance of sustainable low carbon operations and the governance models of the past. The commonality lies in the need to assess projects and prevent risks; the difference lies in the fact that the governance of sustainable low carbon operations is centered on the theme of “green,” including green-related learning, the development of green-themed development strategies, and the development of green behavioral models.

In summary, the following hypotheses are made in this study.

  Hd1: Sustainable operational governance has a positive effect on sustainable low-carbon operations.
  Hd2: Sustainable operational governance has a positive effect on sustainable economic effects.

## 3. Materials and Methods

This section may be divided into subheadings. It should provide a concise and precise description of the experimental results, their interpretation, as well as the experimental conclusions that can be drawn.

### 3.1. Research Model Design

Based on the contents of the literature review and the research hypotheses and objectives of the study, we have constructed a model of the link between corporate culture and sustainable operations in transport infrastructure, as shown in Figure 1.

### 3.2. Questionnaire Design

The study was based on a hypothesis model, and a questionnaire on the interaction between corporate culture and sustainable operational risk was designed through group discussions, expert interviews, and on-site collection. The survey was first conducted in Hunan Province, and the questionnaire was adjusted and improved in response to the pre-survey results so that it could more comprehensively and correctly reflect the subjective views of the respondents. The formal survey contained five latent variables, including Corporate Values (CV), Corporate Culture Management Competence (CMC), Sustainable Economic Effects (SEE), Sustainable Operational Governance (SOG), and Sustainable Low Carbon Operations (SC0) (see Table 1), with each latent variable consisting of four observed variables. The scale was modified from existing literature to ensure its validity of the scale. The questionnaire was measured using a 5-point scale (1 = strongly disagree, 2 = disagree, 3 = no opinion, 4 = agree, 5 = strongly agree). The questionnaire also investigated personal characteristics of gender, occupation, years of experience, and job title level to ensure the validity of the findings. A total of 28 questions were included in the questionnaire.

### 3.3. Data Collection

Hunan Province has a good environment for the development of corporate culture and leading international companies and research universities in the construction, operation, and management of transport infrastructure, so the survey chose the above-mentioned provincial committee as the study area. From 2020 to January 2022, the research team conducted a formal survey of transport infrastructure-related enterprises in Hunan Province and Hubei Province, with questionnaires collected through both field and online surveys. A total of 380 questionnaires were returned, of which 351 were valid, with an effective rate of 92.36%.

The occupational distribution of the respondents was as expected, with 21.08% of middle and senior managers, 52.43% of basic employees, 5.7% of research scholars, and 20.8% of government departments; 7.69% of the respondents held senior titles and 35.33% held associate titles. The distribution of titles in the sample is basically the same as that of the surveyed group; the maximum number of working years is 33.9% within 5 years, and the distribution of working years in enterprises is more even. The software used in the data collation process of this study was SPSS AU. The structure of the researched population of the sample is shown in Table 2.

### 3.4. Methods

In this study, structural equation modeling (SEM), almost from its very beginning, has been divided between covariance-based SEM and composite-based SEM [44–46]. Currently, the commonly used structural equation modeling methods include covariance-based structural equation modeling (CB-SEM) and partial least squares structural equation modeling (PLS-SEM) [47]. In the early years of research, far more articles were published using CB-SEM than PLS-SEM, but after 2015, the number of PLS-SEM-based studies increased rapidly [33, 48]. Currently, PLS-SEM is widely used in the fields of organizational management, business management, international management, and operations management [37, 47, 49, 50].

Both methods have their limitations and applicability. Partial least squares SEM (PLS-SEM), was conceived as an alternate means for accomplishing the same goal as the CB-SEM approach, with advantages in some instances, but disadvantages in situations where the necessary conditions supporting the optimal properties of the CB-SEM approach could be expected to hold [47, 51].

Meanwhile, Hair et al. state that researchers should use PLS-SEM models for research when the research analysis involves testing theoretical frameworks from a predictive perspective; when the current complexity is met by exploring established theories; and when minority groups limit the sample size (for firm-specific studies). This is much less the case with PLS-SEM [52] unlike CB-SEM which strongly relies on the concept of model fit. Therefore, the characteristics of this study were integrated and the partial least squares structural equation modeling (PLS-SEM) was used for the study.

## 4. Result

The analytical process of the study was calculated using the methodology suggested by Anderson, where the strategy model was first evaluated, and based on which the direct linkage of potential variables was analyzed. The software used for data analysis was SmartPLS, developed by Ringle.

### 4.1. Measurement Models

In the PLS-SEM model, the measurement model is analyzed with a primary focus on the analysis of model reliability. scholars have questioned whether the concept of model fit, as applied in the context of CB-SEM research, is of value to PLS-SEM applications in general. Examples of Good-to-fit measures suggested in PLS-SEM models include the standardized root mean square residual (SRMR) and the canonical fit index (NFI; also known as the Bentler-Bonett index) [53, 54]. However, it is important to note that the goodness-of-fit criterion proposed by Hair et al. does not represent a valid measure of model fit [48]. Therefore, in this study, the evaluation metrics were determined by referring to Shmueli et al. and the smart pls manual [55].

By judging the model Good-to-fit (see Table 3), it can be found that the SRMR and NFI metrics of the model meet the requirements and no further adjustment of the model is needed.

In the PLS-SEM model, the measurement model is analyzed with the main focus on the analysis of the model reliability. The reliability tests in this study use: Cronbach's *α*, Composite Reliability, and Factor Loading. Based on Nunnally's study, it can be concluded that in exploratory studies when the Cronbach's *α* value is greater than 0.7 the test is highly reliable. Composite reliability is another important indicator for evaluating the reliability of a model, which usually requires a CR greater than 0.7. As shown in the indicator system of the PLS analysis model in Table 4, Cronbach's *α* values of the measurement models are all greater than 0.7, while the composite reliability values also meet the requirements, so the measurement models have good reliability.

In general, all Factor loading is greater than 0.5 to reasonably explain the latent variables (Barclay, Higgins, and Thompson, 1995), and it can be seen from Table 4 that all Factor loading in this study meets the structural validity requirements. Also, the variance inflation factor (VIF) for all indicators of the model is less than 5, which satisfies the requirements and does not require further adjustment of the model [56]. In addition, the PLS model convergent validity and discriminant validity are mainly based on average variance extracted, which requires AVE to be greater than 0.5 and the square root of the AVE value to be greater than the correlation coefficient of other latent variables. can explain the latent variables better. As shown in Tables 5 and 6, the study data satisfy the above conditions, indicating that there is a good linear equivalence between the measured and latent variables, and the measured variables can explain the latent variables better.

### 4.2. Model Predictive Capability

In PLS-SEM models, *R*^2^ (predicted effect value) and *Q*^2^ (predicted correlation) are commonly used to evaluate the predictive ability of the model. In general, *R*^2^ is weak in explaining power between 0.25–0.5 and moderate between 0.5–0.75, and in this study, *R*^2^ was 0.453, which is generally in line with the requirements. The four endogenous latent variables in the model have a *Q*^2^ of between 0.216–0.337, which meets the requirement of being greater than zero, indicating that the structural model is valid. In addition, according to the Goodness of Fit (GOF) formula, if the GOF value is greater than 0.26, the model is considered to have good applicability in the field of humanities and social sciences. In this study, GOF = 0.4473, indicating that the model fits well.

### 4.3. Model Predictive Capability

As shown in Table 7 and Figure 2, the path coefficients of corporate values on cultural management capability, sustainable low carbon operation and sustainable operational management are 0.569 (*t* = 14.020 > 1.96), 0.199 (*t* = 3.422 > 1.96) and 0.541 (*t* = 13.481 > 1.96) respectively, indicating that hypothesis 1, hypothesis 2 and hypothesis 3 are valid. It also indicates that corporate values have a greater influence on the impact of corporate values on the cultural management capability of a company is significant and has a direct impact on the sustainable management of the company's operations and ultimately whether the company can achieve sustainable low carbon operations. The path coefficients of cultural management capability on sustainable low carbon operation and sustainable economic effects are 0.178 (*t* = 3.122 > 1.96) and 0.230 (*t* = 4.314 > 1.96) respectively, indicating that hypothesis 4 and hypothesis 5 are valid, and the cultural management capability of the enterprise has a certain influence on sustainable low carbon operation and sustainable economic benefit. The sustainable low carbon operation's path coefficient is 0.244 (*t* = 4.234 > 1.96), indicating that sustainable economic effect determines to some extent whether sustainable low carbon operation can be achieved; hypothesis 6 holds; the path coefficient of sustainable operational governance on sustainable low carbon operation and sustainable economic effect is 0.255 (*t* = 3.997 > 1.96), 0.431 (*t* = 14.020 > 1.96), indicating that hypothesis 7, and hypothesis 8 are valid.

## 5. Discussion

In this study, corporate culture is divided into two parts: corporate values and corporate cultural management capability. The sustainable operation of transport infrastructure is divided into three parts: sustainable economic effect, sustainable operational governance machine, and sustainable low-carbon operation, and the influence path of corporate culture on sustainable operation capability is studied, and the hypotheses in the study are confirmed.

1. At the level of corporate values, it can be found through the study that whether a company has mature and reasonable values plays an important role in influencing the cultural management capability of the company. At the same time, corporate values play an important role in a company's ability to govern sustainable operations. Whether or not a company has green and low-carbon values determines whether or not it will choose the appropriate operational strategy in the course of its operations and consciously establish a green and low-carbon brand image in its operations and prevent being labeled as unegree by social media to avoid invisible losses [33]. Therefore, if an enterprise wants to achieve sustainable operations and achieve consensus within the enterprise, it needs to build the direction of its development from the level of its corporate values. At the same time, although the adoption of low-carbon and sustainable operation strategies may have some impact on the development as well as the production capacity of transport infrastructure enterprises in the short term, it has a greater role in promoting the long-term development and long-term economic gains of enterprises.
2. At the level of enterprise cultural management, it can be found through the study that for every 1% increase in an enterprise's cultural management capability, the enterprise's sustainable low-carbon operation capability and sustainable economic effect increase by 0.178% and 0.230% respectively, indicating that the improvement of the enterprise's cultural management capability helps to promote the enterprise's sustainable low-carbon operation capability and economic effect. Strengthening the enterprise's own cultural construction ability and the enterprise's ability to promote its own culture is conducive to improving the management ability of transport infrastructure enterprises and promoting cultural innovation and migration, and forming a corporate culture management model that is more in line with sustainable development and market requirements, which leads to higher economic benefits in the competition.
3. For every 1% increase in sustainable economic effect, the sustainable low-carbon operation capability of the enterprise increases by 0.244%. It shows that whether an enterprise can adhere to sustainable low-carbon operation depends to a large extent on whether it can obtain sufficient economic benefits from the sustainable low-carbon operation. The rationality of this path is that although corporate culture has a significant impact on a company's business strategy, whether a business strategy can be implemented is more absolutely related to the economic benefits of a strategy and whether the strategy is accepted by society. Sustainable and stable economic benefits can provide sustainable and low-carbon operating models for enterprises, and promote their further development from the material level. In addition, ideal social recognition is the invisible benefit of enterprises, which can help enterprises get more opportunities in the exploration of sustainable and low-carbon operating models.
4. It can be found from the study that for every 1% increase in sustainable operational governance capability, the sustainable low carbon operation and sustainable economic effect increase by 0.225% and 0.431%, respectively. This indicates that the sustainable governance capability of an enterprise has an important impact on the sustainable economic effect of the enterprise. Outstanding sustainable governance capabilities can help enterprises minimize the economic and production capacity losses caused by the transformation of sustainable low-carbon operation, avoid risks, and promote sustainable low-carbon operation to produce economic effects and social value more quickly, and to a certain extent also influences whether the enterprise can achieve sustainable low-carbon operation.

## 6. Conclusion

### 6.1. Theoretical Contributions

Previous research on corporate low carbon sustainability has mostly used different theories to explain the influencing factors affecting various aspects of corporate low carbon sustainability, but less literature has focused on the impact of corporate low carbon, sustainability culture, and cultural management capabilities on the effects of corporate low carbon sustainability. In this study, we use corporate culture as a basis for the theoretical expansion of the impact of low-carbon sustainability. The sustainable culture and good cultural management ability of enterprises are important influencing factors on whether enterprises can achieve sustainable low-carbon development, which also implies that the establishment of a sustainable low-carbon development culture and the enhancement of cultural management ability by enterprise managers can help improve the enterprise's ability to manage risks and promote the sustainable low-carbon development of enterprises.

In addition, the conceptual model will also explore for the first time the influencing factors for achieving sustainable low-carbon operations in transportation infrastructure enterprises, for which no relevant studies have been found in the literature. These influences are significant and contribute to the sustainable low-carbon operation of transportation infrastructure enterprises. These findings represent an important original power share of the study.

Another important power share of the thesis is that it explores the relationship between corporate culture and corporate cultural management capabilities, and that good corporate culture can drive the improvement of corporate cultural management capabilities, and this finding also represents a powerful management share that provides a new realization path for companies to improve their cultural management capabilities.

### 6.2. Management Recommendations

1. The implementation of low-carbon management in enterprises is a major trend and a national policy direction in China, and in the case of transport infrastructure enterprises, an essential consumer demand. In an external environment that emphasizes sustainable development, managers need to realize the low-carbon sustainable development of enterprises through the control of corporate culture. At the same time, enterprises, as an important theme of China's national economic system, can only promote sustainable low-carbon development of the whole society if they achieve sustainable development.
2. In the process of realizing the sustainable low-carbon development goals of enterprises, the construction of corporate cultural goals should be emphasized.
3. At the same time, when transport infrastructure enterprises may encounter problems in the process of low-carbon sustainable management that cannot be solved by themselves and market mechanisms, if the market alone operates without the promotion of policy mechanisms, enterprises will lack the motivation to apply technical and management measures that do not have obvious short-term benefits. Therefore, in response to the above-mentioned realities, the government should focus on building a complete policy framework mechanism, constructing perfect subsidy measures, realizing the mutual cooperation between administrative means and market mechanisms, and ultimately realizing the synergistic development between policy formulation and enterprise development to promote the low-carbon sustainable development of transport infrastructure enterprises.

### 6.3. Research Limitations and Future Work

The study has some limitations that should be considered in future research. The survey group in this study focused on one country, so whether the findings can be generalized to the remaining social contexts requires further research. Therefore, future research should focus on investigating the adaptability of the model to the remaining cultural regions. The adaptability of the model can be improved in the future by increasing the scope of the survey to include consideration of different regional cultures.

Another limitation of this study is that the scope of the study is limited to transportation infrastructure-related enterprises, and the adaptability of the findings is somewhat lacking. The scope of the research can be expanded in future studies to enhance the adaptability of the findings.

## Figures and Tables

**Figure 1:** Research model.

**Figure 2:** Structural model.

**Table 1:** Statistics on latent and observed variables.

Latent variable	Observed variable
Corporate values	Social responsibility
	Values alignment
	Shared vision
	Innovation orientation
Corporate culture management capabilities	Cultural innovation
	Cultural management model
	Cultural migration
	Willingness to accept culture
Sustainable economic impact	Market orientation of metro behaviour
	Government subsidies
	Long-term cost savings
	Green transition inputs
Sustainable operational governance	Risk prevention
	Green exploration
	Green strategy
	Green behaviour
Sustainable low-carbon operation	Green dynamic capabilities
	Green product development
	Green innovation
	Carbon reduction capability

**Table 2:** Structure of the surveyed population.

Variables	Type	Value	Proportion (%)
Gender	Male	176	50.14
	Female	175	49.86
Occupation	Corporate senior management	23	6.55
	Middle management	51	14.53
	Enterprise grassroots staff	136	38.75
	Government departments	73	20.8
	Researchers and academics	20	5.7
	Others	48	13.68
Title level	Full senior title	27	7.69
	Associate title	124	35.33
	Intermediate title	113	32.19
	Junior and below	87	24.79
Years of work	<5	119	33.9
	5–10	83	23.65
	10–15	89	25.36
	>15	60	17.09

**Table 3:** Good-to-fit table.

Indicator	Value	Judgment criteria
SRMR	0.066	<0.08
NFI	0.917	>0.9

**Table 4:** Indicator system for PLS analysis model.

Latent variable	Cronbach`s *α*	Composite reliability	Factor loading	*t*-test	VIF	Explicit variable indicators
Corporate values	0.891	0.925	0.835	28.341	2.291	CV1
			0.872	30.025	2.651	CV2
			0.827	31.222	2.031	CV3
			0.939	33.764	4.134	CV4
Corporate culture management capabilities	0.881	0.918	0.861	30.394	2.257	CMC1
			0.898	31.335	2.112	CMC2
			0.842	31.892	2.044	CMC3
			0.831	30.935	2.727	CMC4
Sustainable economic impact	0.888	0.922	0.838	32.159	2.06	SEE1
			0.854	31.707	2.289	SEE2
			0.862	32.493	2.321	SEE3
			0.905	33.163	2.97	SEE4
Sustainable operational governance	0.889	0.924	0.853	29.200	2.327	SOG1
			0.853	29.916	2.328	SOG2
			0.832	33.411	2.074	SOG3
			0.927	30.681	3.534	SOG4
Sustainable low carbon operation	0.891	0.925	0.864	31.518	2.426	SC01
			0.846	30.888	2.196	SC02
			0.853	30.253	2.182	SC03
			0.910	31.239	3.097	SC04

**Table 5:** Latent variable AVE values.

Latent variables	Average variance extracted
Corporate values	0.755
Corporate culture management capabilities	0.737
Sustainable economic effects	0.748
Sustainable operational governance	0.752
Sustainable low-carbon operation	0.755

**Table 6:** Correlation coefficients between AVE square root and latent variables.

Latent variables	Corporate values	Corporate culture management capabilities	Sustainable economic effects	Sustainable operational governance	Sustainable low-carbon operation
Corporate values	0.869				
Corporate culture management capabilities	0.569	0.859			
Sustainable economic effects	0.544	0.502	0.869		
Sustainable operational governance	0.503	0.434	0.542	0.865	
Sustainable low-carbon operation	0.541	0.472	0.548	0.540	0.867

**Table 7:** Description of model hypothesis testing results.

Hypothesis	Relationship	Path coefficient	*T*-value test	*P*-value test	Results
Ha1	CMC-> SC0	0.178	3.122	0.002	Accept
Ha2	CMC ->SEE	0.230	4.314	<0.001	Accept
Hb3	CV ->CMC	0.569	14.020	<0.001	Accept
Hb1	CV ->SC0	0.199	3.422	0.001	Accept
Hb2	CV ->SOG	0.541	13.481	<0.001	Accept
Hc	SEE ->SC0	0.244	4.234	<0.001	Accept
Hd1	SOG ->SC0	0.225	3.997	<0.001	Accept
Hd2	SOG ->SEE	0.431	14.020	<0.001	Accept

## Data Availability

The raw data supporting the conclusions of this article will be made available by the authors without undue reservation.
